The article "Deep Learning in Healthcare System for Quality of Service" was retracted in 2023. Reasons: signs of a paper mill; suspected computer-generated content; unreliable results or conclusions; concerns about the data.

# Deep Learning in Healthcare System for Quality of Service

**DOI:** 10.1155/2022/8169203

**Published:** 2022-03-08

**Authors:** Dibyahash Bordoloi, Vijay Singh, Sumaya Sanober, Seyed Mohamed Buhari, Javed Ahmed Ujjan, Rajasekhar Boddu

**Affiliations:** ^1^Department of Computer Science and Engineering, Graphic Era University, Dehradun, Uttarakhand, India; ^2^Prince Sattam Bin Abdul Aziz University, Wadi Al Dawasir 1191, Saudi Arabia; ^3^Department of Information Technology, King Abdulaziz University, PO Box 80221, Jeddah 21589, Saudi Arabia; ^4^Department of Zoology, Shah Abdul Latif University Khairpur, Khairpur, Sindh, Pakistan; ^5^College of Animal Sciences and Technology, Northwest A and F University, Xianyang, China; ^6^Department of Software Engineering, College of Computing and Informatics, Haramaya University, Dire Dawa, Ethiopia

## Abstract

Deep learning (DL) and machine learning (ML) have a pivotal role in logistic supply chain management and smart manufacturing with proven records. The ability to handle large complex data with minimal human intervention made DL and ML a success in the healthcare systems. In the present healthcare system, the implementation of ML and DL is extensive to achieve a higher quality of service and quality of health to patients, doctors, and healthcare professionals. ML and DL were found to be effective in disease diagnosis, acute disease detection, image analysis, drug discovery, drug delivery, and smart health monitoring. This work presents a state-of-the-art review on the recent advancements in ML and DL and their implementation in the healthcare systems for achieving multi-objective goals. A total of 10 papers have been thoroughly reviewed that presented novel works of ML and DL integration in the healthcare system for achieving various targets. This will help to create reference data that can be useful for future implementation of ML and DL in other sectors of healthcare system.

## 1. Introduction

Industry 5.0 and 5G wireless communication has led to the development of cost-effective sensors, thereby leading to the emergence of Internet of things (IoT). It has an indispensable role in today's healthcare system. Internet of medical things (IoMT) is a crucial component of the modern healthcare system [1]. IoT is an ever-expanding, limitless ecosystem that integrates software, hardware, or any other device equipment that collects or exchanges data. IoT in the healthcare service network is known as IoMT. The need for telemedicine, remote patient monitoring, automated diagnosis, detection, and treatment of acute diseases has become eminent, especially after the COVID-19 pandemic. Monitoring systems in the healthcare business are now possible thanks to Internet of things (IoT)-enabled devices, which can keep patients safe and healthy while also allowing physicians to give better care. Patient engagement and satisfaction have increased as interaction with doctors has become simpler and more efficient. Furthermore, remote monitoring of a patient's health aids in the reduction in hospital visits and the avoidance of readmissions. IoT has a big influence on lowering healthcare expenses and increasing treatment results. The Internet of things (IoT) is clearly transforming the healthcare industry by redefining the role of gadgets and human touch in medical solution delivery [2, 3]. IoMT of wide range is useful in patient conditioning, monitoring, screening, personalized medicine, integrating healthcare professionals, doctors, and hospital networks to patients for remote telemedicines, and patient monitoring. As the IoMT and IoT increase, the data generated by these devices also increase. This substantial amount of data is generally stored and regulated on the cloud servers. Health data are useful in many ways when processed intelligently [4, 5]. The intelligent processing of health data may help to prevent pandemic outbreaks in a city, states, or countries, helping to identify acute diseases such as Alzheimer's disease, diabetes, cardiovascular diseases, and lung cancer [6]. Blockchain is more reliable and robust as once the data are created, it can only be read and not edited or updated. Blockchain also facilitates time stamping along with the use of asymmetric cryptography for secure transactions in the trusted network. In addition to that, it also provides data for the development of DL/ML models. The transactions do not require additional protocols that make blockchain an adaptive nature that can be integrated with different types of data, platforms, and devices. The health data obtained from the electronic health record, genomic sequence, and digital health wearable are so great and cannot be reviewed easily without the intervention of artificial intelligence, deep learning, or artificial neuro-networking [7–9]. ML, DL, and AI have a proven record of demonstrating the capacity to translate large unmanaged data into actionable knowledge in various fields of agriculture, supply chain management, quality control, sales forecast, security, fraud detection, and other major fields.

Deep learning is the part or branch of machine learning. Well with the growing number of machine learning techniques in health care, we can see a future in which data, analysis, and invention collaborate to help countless individuals without their knowledge. Soon, ML-based applications packed with real-time patient data from many healthcare systems across several nations will be ubiquitous, increasing the efficacy of hitherto inaccessible treatment options [10, 11]. Machine algorithm learning is discovered by John McCarthy, and the division of machine learning is discovered by Arthur Samuel. ML and DL are the approaches of AI, where AI can be defined as the artificial creation of a human brain line system that can learn natural language and plan, perceive, and process it for making decisions with minimal intervention of human. Many individuals, organizations, small businesses, and government agencies use ML and DL for complex and diverse data processing and achieving multi-objective goals such as maximizing profit, minimizing production cost, forecasting sales, and improving operational and supply chain management. ML and DL were also found to have an indispensable role in healthcare data management, and the classification of AL, ML, and DL is shown in Figure 1.

With the advancement in the computational system emerge several computing technologies such as artificial intelligence, IoTs, and big data in various fields, especially in healthcare system IoHTs that give the fruitful result to recognizing the daily life activity of diverse wearable devices. The target is achieved by deep learning of HAR in IoHTs. We know the types of deep learning such as supervised, unsupervised, and semisupervised. With the help of semisupervised deep learning, the chances of accurate data related to human activities analyse the considered data fairly to train the classifier data. For the effective accurate results of labelled sample, the intelligent auto-labelled scheme based on deep learning can improve the learning efficiency in IoMTs.

### 1.1. Advantages of DL and ML in Medical Healthcare Data

The deep learning and machine learning are evolutionary changes in various fields such as industry, companies, schools, colleges, and healthcare systems, and we can say that more changes are seen in the medical line by providing many types of online and offline facilities. Deep learning plays an important role in the detection of cancer cells automatically. The ML can be solving multiple tasks but it needs human beings, while the DL performs alone or automatically using machine learning. Deep learning solves the whole problem unlike ML automatically. Deep learning is more beneficial for elders, coma patients, and cardiac disease diagnosis, especially in case of children [12]. The application of AI and other approaches is shown in Figure 2.

Deep learning is beneficial for the recognition of any problem, and the data-driven performance is also better in any type of problem. The learning algorithms are simple, i.e., easily learned or performed and easily able for application. The machine learning is nonlinear, and traditional deep learning is able to make fast and powerful machine learning for language learning and is responsible for accurate patient's data. The representation of patient's information or data in various types, i.e., images and text, can be learned like the real-time condition of the patients [13]. Recent deep learning models for healthcare applications, on the other hand, are sophisticated and need a great amount of computing resources for training and prediction. It also takes a long time to train and evaluate data using these sophisticated neural networks. The more advanced the network and the longer the forecast period, the higher the accuracy required. This has been a significant issue in healthcare and other IoT applications where real-time findings are crucial [14, 15]. The deep learning is gifted to deliver the potential for enhancements in worth control engineering system. Machine learning is responsible to provide beneficial tools for understanding the domain. The ML gives the chances for the examination of the dynamic system and able to change the surroundings and able to recognize the data in different forms of data. With the help of deep learning, the detection of genetic diseases such as Turner's syndrome, hemophilia, and sickle cell anemia can be easily detected by the study of genes and the doctors are able to find the treatments for the future and future medication. The deep learning and machine learning *g* are able to find the normal and abnormal data of the patients, by that the doctors can detect the condition of patients.

Machine learning is also known as artificial intelligence, which is used for recognizing or diagnosing the real-time condition of the patients. The deep learning has the ability to regenerate the real-time condition of the patients on the basis of raw data or from previous data of the patients. Due to this ability, it can be used in various fields such as healthcare system, for security of cybercrime industry. However, it plays a vital role in healthcare system, especially for children and old age elders, and recently, elders are preferred to be alone enduring. By considering the facts, the deep learning is obligatory for the advancement.

In modern time, the fatal rate increases day by day with cardiovascular disease (CD). The children and elders do not prefer the wearable devices due to irritation, and in those cases, deep learning is applied for gathering the data while the wearable devices are having the ability to find or recognize the real-time condition of patients. In this modern era, the acute diseases such as diabetes, Alzheimer's diseases, genetic diseases, cancer, and respiratory malady can be minimized by applying smartness in healthcare system that is possible using computational learning system, SHM, IoT, and knowledgeable doctors who have the capability to detect the real-time condition of the patients and have the proper information or prediction of future condition.

According to the medical survey, there are about 30% of the population suffering from cardiovascular diseases. We can say that the computational learning or robotic learning is used for the smart health monitoring because smart health monitoring is the amalgamation of health monitoring devices and IoT and artificial intelligence. The SHM plays a vital role in the healthcare system in this modern era. Artificial intelligence is applied for the uses of machine learning algorithms and software in healthcare systems. The results of artificial intelligence are based on the data used in machine learning. In essence, this is discovered by the game. The working of deep learning models is based on the convolutional neural network (CNN) learning, because it is a type of artificial neural network (ANN) that is applied for the visualization of images such as ultrasound, MRI, CT scan, and X-ray.

The computational learning is applied in healthcare system when the working of smart health monitoring devices and IoTs is unable to detect the patient's data. These algorithms are able to recognize the behavioral data and form their own models; machine learning is also known as artificial intelligence. It is the method in which the CNN and ANN are able to form an artificial neural system of an animal (AI), and it works in two forms: 1. algorithms are literal and 2. deep learning may be applied in the form of black boxes. Deep learning is working on the basis of linear methods unlike nonlinear traditional method in which the individuals undergo unwanted visits of the hospitals, but now they can be communicated with the doctors computationally.

There are various types of devices that are used for different types of disease monitoring such as accelerometer for the detection of breathing rate, cardiovascular defibrillator, and pacemaker that are used for the diagnosis of breathing rate and blood pressure along with body temperature of the patients, which are the basic parts of IoTs. Deep learning is also useful for the detection of daily life activities, when the whole data are collected using microphone sensor arrays that are working on the basis of two-dimensional spectrum convolutional neural network (DCNN). The daily life activities and behavior of the patients can be detected by many types of wearable and nonwearable devices and also by smart homes that are totally digitalized by fixing the sensors such as toilet seats, smart pillow, smart bed, and smart floor. The behavioral activities are classified into two categories of short-term and long-term activities; short-term activities can be changed from hours to days, such as repeated use of toilet that may be caused by stomach upset, and long-term activities can be changed from a few days to months, or years; in this, the repetition of all activities in a day indicates the memory loss or Alzheimer's disease. The deep learning is more beneficial for the detection and possible treatment of these diseases [16]. The deep learning consists of two phases: 1. training and 2. inferring training, which involves the labelling of large data and identifies the feature. Inferring involves memorization and makes the results on the basis of previous data.

The primary goal of this study was to analyse this relationship by focusing on two types of operational issues. Using real-world examples, here we demonstrate how machine learning can improve human abilities to comprehend and manage healthcare operations, resulting in more efficient health care. While medical computerization and digitalization have made tremendous advances, healthcare management systems have yet to profit greatly from these breakthroughs due to the high complexity and unpredictability of healthcare operations. The author has found that the systematic review of AI, ML, and DL roles in healthcare is lacking in the public domain. This motivates the author to present the review on the recent integration of AI, ML, and DL in various healthcare frameworks for enhancing the quality of service and health of patients. Disease outbreaks and emergence have become a big issue in today's fast-paced world of technology and change. In terms of disease prevention, control, and prevention, technology has become a major issue for healthcare practitioners and healthcare business. Maintaining a healthy lifestyle has become hard due to demanding job schedules. A smart health monitoring system is the solution to the aforementioned issues. The recent industry 5.0 and 5G revolutions have resulted in the development of smart, low-cost sensors that help in the real-time monitoring of people's health. Traditional healthcare systems were unable to provide fast, cost-effective, and trustworthy health monitoring services from remote locations, but the SHM has made it possible. Thus, the author presents a state-of-the-art review of some of the major implementations of AI, ML, and DL in healthcare data for data management, early detection, medication, data security, and detection. AI and machine learning are revolutionizing the healthcare market, as they are in virtually everything else industry. From the possibility of deep learning and neural networks in pharmaceutical research to the increasingly sophisticated use of intelligence diagnostic tests and surgical robotics, AI is changing the way we design cars, optimize our energy usage, and maintain our finances. It is also bringing new opportunities—and risks—to human health management. The ability of AI to bring together huge oceans of data that saturate every aspect of healthcare to improve decision-making between the sector's key stakeholders, from pharmaceutical innovators to healthcare professionals, binds it all together [17, 18].

## 2. Review of Papers

In recent times, the DL and ML have been extensively used in the smart health monitoring network and healthcare services. The DL and ML were used to analyse the health data that are generated by various IoMT devices and sensors. These health data have been stored and handled by cloud network and cloud services. ML and DL are implemented to analyse these complex health data to achieve multi-objective tasks. According to Mohammad Ali et al., there are about 50 billion devices that were added to the medical field by the end of 2020 and face many security challenges. According to him, the DL/ML is also used for gathering big data along with the recognition of threats in cybercrime [19].

In the recent work of Imran Ahmed et al., he has discussed the use of data that are collected through the IP-based RGB camera that is installed at the height of 4 meters and takes the top view of the patients and the data recorded at the Institute of Management Science, Peshawar, and these data are collected for the detection of discomfort of the patients by the movement of patient's body. This camera helps in the detection of the discomfort level of patients. The deep learning algorithms (models) are used for identifying the level of discomfort from the top. The Mask R-CNN 19 is applied to the patients for recognition. These experiments use various kinds of measures for the evaluation such as TPR, FPR, TNR, and MCR, and for the video records, the FDR and TDR are used. The average performance for various organs of the patient body in the videos is summarized and presented in Table 1. It is noticeable that the model was able to detect the discomfort with FPR of 7% and MCR of 4%.

In the healthcare system, we can say that the IoT and SHM play an important role in this field for enhancing the real-life smart applications; i.e., they play a vital role in this time when COVID-19 is established as a pandemic by the World Health Organization, and the detection of coronavirus is difficult in early time of pandemic, but now it can be easily diagnosed using *X*-rays of chest. There are only small images of *X*-rays, CT scan, and MRI, which are detected because COVID-19 is a new disease entered in this era, and the less number of the techniques are used such as Inception V3, Dark Convent, and Convent. In this pandemic era, many researchers are at work on the treatment, diagnosis, and methodology of COVID-19.

According to Hemant Ghayvat, the deep learning is also applied to the daily life activities with the help of various kinds of devices. The recognition of daily life activities is more useful for the elder ones who prefer to survive alone today. Almost about 30% of the total population are above 60 years old who need the proper caretaker and disease-free life. The mortality rate of individuals by acute diseases of these ages can be cured or treated by applying smartness in the healthcare system. This is done by the use of smart health devices such as smartphones and global poisoning system (GPS), and this is more suitable for recognizing outdoor activities. At the present time, the spatial and other information is collected using the convolutional neural network (CNN). The acoustic-based monitoring system does not show excellent results due to security issues. The identification of daily life activities involves three stages, and at first stage, the data are collected by the daily exercises, and spread on the bandwidth capacity is shifted by the channels that are inclined by the physical exercises and by recorded data. With this method, the collected data are right or accurate, and this procedure uses online methods for the recording [20]. Hemant's model is found with 90% and 83% accuracy during testing and training, whereas the loss was 0.5% and 1% for testing and training. The accuracy of various activities along with performance graph is presented in Figures 3 and 4.

The framework that is used for the smart health monitor is the combination of compressed sensing (CS), machine learning-based models, ADMM, and the binary CNN classifier. Abrar Zahin works on the convolutional learning that it works or records accurately and works with proficiency. In this study, the researcher uses the terms ADMM and CS, which are helpful in simplifying the software. The wireless camera nodes are used for collecting large amounts of images. Then, these images are transferred to the main processing center, and here, any changes in health are detected [21]; the author selected the 597 cases with 14 features such as age, sex, chest pain type, resting blood pressure, cholesterol, number of smoking years, and blood sugar levels. The best accuracy of the proposed model was found to be 84% and was higher than other regression naive Bayes and decision tree models. The model accuracy peaked at 98.5% when the proposed feature selection weighting methods were applied for the detection of heart diseases as shown in Figure 5.

Shresth Tuli et al. discuss the health fog; it is a method of detection of heart diseases with the help of deep learning, and it collects the patient's data using fog bus framework. The health fog models are based on IoT, which can manage the data effectively and able to diagnose the seriousness of patients. The healthcare system is a vast project. The researchers are focused on the edition of health fog in the healthcare system for automatic diagnosis of acute heart diseases using deep learning and IoT devices. The fog is able to manage the data that are collected from different IoT devices. The predictions of heart patients with fog systems are much accurate compared with the prior system that lacks the utilization of deep learning and IoT, and hence, the results were inaccurate and insufficient for the records and the models that are based on deep learning are highly accurate. They used the fog bus framework in their work for the detection of real-time conditions of heart patients. The health fog system is now applicable for other health domains such as diabetes, cancer, hepatitis, genetic diseases, and genetic disorders. Fog system is open-source software [14]. It was found that the proposed mode training accuracy increases and test accuracy decreases with increasing number of nodes. Increasing nodes increases the training data and decreases the test data subset. The prediction accuracy increased by 16% with the implementation of DL in the existing framework. The performance characteristics of the proposed model are presented in Figure 6, indicating higher accuracy, lower latency, and low power consumption.

The wireless body sensor network (WBSN) [22] also has a great role in healthcare system that helps in the detection of the real-time condition. The WBSN faces major challenges such as feasible discussion in emergency cases, and these challenges are overcome using fractional cat-based scalp swarm algorithms (FCSSA). It records the whole data using several types of parameters, and WBSN is used to transfer the data to the target node and then returns it back to the target node. The hybrid harmony search algorithm and practical swarm optimization (hybrid HAS-PSO) are used for the determination that forms the results, and here, the deep belief network (DBN) classifies the whole data for the assessment. The FCSSA works in a better way with matrices of 94.604 accuracy, 0.145 energy, and 0.058 throughput values. The performance parameters were compared with existing models, namely low-energy adaptive clustering hierarchy (LEACH), particle swarm optimization (PSO), and artificial bee colony (ABC) for three data sets from Cleveland, Hungary, and Switzerland. It was found that the integration of DL in the proposed framework led to the highest accuracy of 94.6% along with the least energy consumption and highest throughput for all data sets when compared to the competing models. The summarized results are presented in Figure 7.

Heart disease and cardiovascular diseases (CD) increase the mortality rate, and the cases of heart attacks, heart stroke, and brain stroke are more compared with others, which are prevented by the use of deep learning modified neural network (DLMNN) because it can detect the heart diseases at initial stages and helps in future medication. The DLMNN is implemented by the three steps including (1) authentication, (2) encryption, and (3) classification. In the first step, the substitution cipher and SHA 12 are collectively used, which are helpful for the authentication of heart patients from different hospitals. The wearable devices that fixed into the patient's body by the patient collect the actual data and transfer it to the cloud. Now, the censored data are securely transmitted using the PDH-AES technique. Here, the encrypted data are now decrypted. After this, the whole data undergo classification by the DLMNN classifier. The classified final data may be normal or abnormal and show the condition of the patients [23]. The PDH-AES is 95.8% able to secure the whole data, so the security cannot be found.

According to a recent study, the cases of Alzheimer's disease (AD) are increasing day by day, and there may be up to 60% to 70% cases that can be seen in the age of 20 to 30 years. Alzheimer's disease is a neurologic disorder that affects the brain to shrink (loss of function) and brain cells to die. The most common kind of dementia is Alzheimer's disease, which is characterized as a gradual loss of cognitive, behavioral, and social abilities that limit a person's ability to function independently. One of the earliest signs of Alzheimer's disease is forgetting recent events or talks [24, 25]. As Alzheimer's disease progresses, a person's memory will deteriorate and he or she will lose the ability to do daily tasks. The cases with mild cognitive impairment (MCI) disease are less than AD, a highly heterogeneous phenotypic spectrum. There are almost about 10 to 20% of MCI growths to AD, and this is a gradual process but does not take much time more than a year; hence, it is difficult to identify the progression, and the way of conversion to AD from stable MCI can be identified with the help of deep learning. The ML and DL play an important role in the diagnosis of AD. The patient's data are heterogeneous in nature, which involves data from magnetic resonance imaging (MRI), positron emission tomography (PIT), X-ray, CT scan, etc. Alzheimer's disease models are based on the CNN and single MRI images, but these data are not accurate and do not give proper information about the real-time condition of the patients, and hence, the advanced deep learning is applied and multimodal data are used. These models are based on the five time-series modalities and CNN-BiLSTM design, which can give great results that help improving the monitoring of Alzheimer's diseases [26].

The smart healthcare system is the solution for widely spread acute diseases towards the old age population. SHM monitors noncommunicable lethal diseases in elders by observing daily life activities. There are many more challenges in front of this smartness in healthcare systems such as remote monitoring environment, communication technologies of this environment, and presence of intelligence processing system. There are many smart sensors and smartphones used for human activity recognition (HAR) algorithms. The sensors are fixed in smart devices and wearable devices such as smartphones, Fitbit watches, and hand bands that are able to recognize every activity of an individual such as walking, running upstairs by measuring blood pressure, respiratory rate, and fitness tracking. There are some drawbacks observed in these devices, i.e., the inaccuracy of data acquisition [R]; it is needed for high computational system. The accuracy and classification efficiency can be improved by the addition of group-based context of human activity recognition (GCHAR). The GCHAR is structured in two-level hierarchical groups such as intergroup and inner group. The accuracy of HAR is improved by the GCHAR, and it is proved by the experimental comparison with the other algorithms as shown in Figure 8.

It is worthwhile to note that GCHAR algorithms outperform the other algorithms by a good margin as shown in Figure 8. The higher accuracy of 94.16% is achieved by this algorithm. The accuracy of the algorithm is based on two aspects such as the hierarchical classifier structure able to reduce the misclassification and inaccuracy. Secondly, the error correction utilization of context awareness improves the correction measurement and whole performance [27].

The routine HAR can be improved using various types of algorithms and compared among these algorithms to recognize the betterment. For the experiment, the researcher selects the minimum eight human activities denoted by *A_s_A*_1,_*A*_2,_*A*_3,_ and on and along with classifying *C*_1_, *C*_2_, *C*_3_,...., so on. For the demonstration of all activities, we can use the receiver operating characteristic (ROC) curves, which are shown in Figure 9. The eight solid lines show the different human activities (HAs) in which the average value of the area under the curve (AUC) is 0.95. According to the figure, the *A*_1_ activity obtains the best performance and the *A*_5_ shows the worst performance. For the comparison among the performances of these activities, we can use some other kinds of algorithms such as DNN, SVM, and RF for the improvement as shown in the next figure. In this figure, when the AUC value is 0.95, all three algorithms can only achieve the values of 0.87, 0.74, and 0.90, respectively. The reason for these values and position of activities in the figure is that the on-body positions form exclusive data for the accuracy than the other positions [28].

Deep learning and machine learning play an important role in diabetic patients for the prevention of readmission in hospitals. According to researchers, the diabetic patients are widely spread all over world. The number of people with diabetes increases from 1980, i.e., 180 million to 422 million in 2014. Type 2 diabetes is more spread in underdeveloped countries around 17.1% in 2004, and it increases 30% in the last ten years. This can be done by the combination of convolutional neural network (CNN) and data engineering that works as outbreaks from other algorithms. It has been found from Figure 10 that the integration of deep learning methods in the existing frameworks leads to improvement in accuracy F1 and area under curve parameters in identifying the diabetic patients [29].

### 2.1. Disadvantages and Future Challenges

The deep learning and machine learning are the main reason for the advancement in the medical field, but there are some limitations that can be seen like it needs the huge data for recognition and for making results, which are impossible sometimes. With the bulky data, it may be complex and forms complex data models, and hence, these computational techniques are more expensive. Therefore, this is unable to apply for everyone, and hence, they cannot take the proper benefits of this technique. Deep learning: the deep learning is more prone to error chances of errors that are occurred in training and testing of data due to bulk of data. Sometimes data become inconsistent, and this is due to continue updating.

No doubt the robotic learning or ML/DL plays a more important role in every field, but there are some challenges that are faced by it. First of all, this type of learning lacks interpretability, requires bulky data, is sometimes unable to handle the direct symbols and decision-making support, and has difficulty in dealing with natural languages. The deep learning methods require a large amount of data; hence, the handling of the data is much difficult and consumes more time and storage. The study of deep learning methods can only understand by those doctors or medical individuals who is having the proper knowledge of linguistic grammar and patient's health data.

### 2.2. Security Issues in ML/DL

IoT devices used a lightweight framework, thus prone to denial of service (DoS), jamming, spoofing, man-in-in-the-the-middle software attacks, and privacy leakage. Sybil and spoofing attacks are also common. Many ML/DL-based frameworks are available in the public domain for security. ML/DL-based authentication, access control, secure offloading, and malware detection models are available but lack speed and accuracy at the early learning stage, high computation, and communication cost along with the risk of unsupervised learning. Different types of IoT have many organizations that form the security standards, and the organizations are IEEE and ETSI, because they are able to form security norms. A big IoT system needs the higher and robust security such as blockchain technology [30, 31]. The ML/DL of security of IoTs is categorized into IoT system, IoT threats, and learning method for IoT security/DL security. On the basis of IoT security learning, ML approaches include supervised approaches, unsupervised approaches, semi-supervised approaches, and RL methods [32]. The DL learning is also differentiated into supervised, unsupervised, and semi-supervised.

## 3. Conclusion and Future Scope

The present work shows the integration of ML and DL in healthcare system for various applications, namely disease-discomfort detection, diagnosing cancer, diabetes, tumor, respiratory malady such as acute diseases, and prevention of outbreak of pandemic or endemic diseases in a particular region city or state. The recent developments in the ML/DL models and framework have shown remarkable performance in the IoMT network and services. ML/DL also showed the proven record in clinical decision-making capabilities under supervised conditions. The use of ML and DL is essential to get useful information from complex and considerable health data generated by the healthcare systems in terms of electronic health record, medical images, ECG, EEG records, and data obtained from real-time health monitoring wearable devices and sensors. The present work will help to generate ideas for future implementation of ML and DL in other aspects of the healthcare system. However, the present work in not including much about the role of ML and DL in the security system of healthcare frameworks is a vast and complex domain. The author considers the review of such work as a future plan.

## Figures and Tables

**Figure 1:** Classification and subclasses of AI, ML, and DL.

**Figure 2:** Applications of ML and DL in the healthcare system.

**Figure 3:** Accuracy performance of the model during training and testing on data.

**Figure 4:** Loss performance of the model during training and testing on data.

**Figure 5:** Comparison of classifier accuracy of the proposed model with existing similar models for different number of features in the set.

**Figure 6:** Training and test accuracy with different number of nodes.

**Figure 7:** Comparison of performance parameters of the proposed model with the existing model for different sizes of data set.

**Figure 8:** Comparative evaluation of classification accuracy among GCHAR and related classification algorithms.

**Figure 9:** (a) Comparative result of the activated various algorithms and (b) class-wise performance of the proposed model.

**Figure 10:** Comparative results of performance parameters before and after implementation of deep learning algorithm in the existing framework.

**Table 1:** Performance parameters for all organs of the patient in video.

Average performance	Head	Right arm	Left arm	Right leg	Left leg	Torso	Average
Accuracy	92	93	93	93	94	94	94
MCR	7	4	3	4	4	4	4
TPR	92	93	93	93	93	94	94
FPR	9	8	6	8	7	5	7
TNR	90	91	90	91	90	92	91

## Data Availability

The data pertaining to this article are included within the article.
